# LCC-Net: A Lightweight Cross-Consistency Network for Semisupervised Cardiac MR Image Segmentation

**DOI:** 10.1155/2021/9960199

**Published:** 2021-05-17

**Authors:** Lai Song, Jiajin Yi, Jialin Peng

**Affiliations:** ^1^College of Computer Science and Technology, Huaqiao University, Xiamen 361021, China; ^2^Xiamen Key Laboratory of Computer Vision and Pattern Recognition, Huaqiao University, Xiamen 361021, China

## Abstract

Semantic segmentation plays a crucial role in cardiac magnetic resonance (MR) image analysis. Although supervised deep learning methods have made significant performance improvements, they highly rely on a large amount of pixel-wise annotated data, which are often unavailable in clinical practices. Besides, top-performing methods usually have a vast number of parameters, which result in high computation complexity for model training and testing. This study addresses cardiac image segmentation in scenarios where few labeled data are available with a lightweight cross-consistency network named LCC-Net. Specifically, to reduce the risk of overfitting on small labeled datasets, we substitute computationally intensive standard convolutions with a lightweight module. To leverage plenty of unlabeled data, we introduce extreme consistency learning, which enforces equivariant constraints on the predictions of different perturbed versions of the input image. Cutting and mixing different training images, as an extreme perturbation on both the labeled and unlabeled data, are utilized to enhance the robust representation learning. Extensive comparisons demonstrate that the proposed model shows promising performance with high annotation- and computation-efficiency. With only two annotated subjects for model training, the LCC-Net obtains a performance gain of 14.4% in the mean Dice over the baseline U-Net trained from scratch.

## 1. Introduction

Medical image analysis plays an increasingly important role in routine clinical work. Magnetic resonance imaging (MRI) is a noninvasive technique for investigating cardiac structures, thus widely used in clinical diagnosis and treatment. Segmentation of the left ventricle (LV), right ventricle (RV), and the myocardium (MYO) from cardiac MR images can provide crucial diagnostic parameters about the cardiac. Recently, convolutional neural networks (CNNs), mostly fully convolutional networks (FCNs) [1, 2], have made substantial progress for cardiac image segmentation [3]. However, the current supervised-learning models rely heavily on a large amount of manually labeled data for model training to achieve competitive performance. Unfortunately, manually labeling cardiac MR images is time-consuming and labor-intensive and requires strong domain knowledge from experts. Moreover, most of the top-performing methods are deep and wide convolutional neural networks involving a massive number of training parameters, which not only increases the chance of overfitting but also hinders their applications in clinical routines. To address the above problems, we introduce a lightweight deep network for semisupervised segmentation of cardiac images. Our model is trained only on a few labeled subjects and a more considerable number of unlabeled subjects.

There are generally two paradigms to make use of unlabeled data. The first one is unsupervised or self-supervised pretraining, followed by fine-tuning on a small set of labeled data. The second paradigm is to jointly use the labeled data and unlabeled data through pseudo labeling [4] or consistency regularization [5–8]. Since there is an obvious gap between the objectives of the unsupervised pretraining and the downstream segmentation, the effect of unsupervised pretraining is not always significant. In this study, we follow the second paradigm and make use of the unlabeled data by enforcing consistency regularization on the supervised model, aiming to improve the generalization ability of the supervised trained model and reduce the risk of overfitting. Consistency regularization encourages the segmentation prediction to be consistent on the unlabeled examples under different data perturbations or among different models. We follow the studies in [6, 9, 10] and enforce consistency among different models' predictions. Both strong and weak perturbations are applied.

In this study, we propose a lightweight network, LCC-Net, for semisupervised segmentation of cardiac MR images based on consistency training cross models. To be specific, our model, as shown in Figure 1, consists of one shared encoder and three separate decoders: one decoder for supervised learning and the other two decoders for unsupervised consistency learning. Following a similar strategy as in [6], different perturbations are injected on the two unsupervised decoders. We enforce consistency between the predictions of the supervised decoder and unsupervised decoders to make the learned model less sensitive to the extra perturbation. To further improve model robustness and reduce the risk of overfitting, we augment the input data, both the labeled and unlabeled data, with extreme perturbations realizing significant gains. While the previous semisupervised models suffer from a massive scale of parameters and high computational complexity, we lighten our model with the lightweight Ghost module introduced in [11]. Moreover, we validate the proposed method on the ACDC [12] dataset.

The rest of the paper is organized as follows. In Section 2, we briefly review the related work.  Section 3 presents the proposed method, which is evaluated on challenging cardiac segmentation tasks in Section 4.  Section 5 concludes this study.

## 2. Related Work

### 2.1. Cardiac MR Image Segmentation Methods

For cardiac MR image segmentation, Painchaud et al. [13] presented a postprocessing VAE [14], which converts anatomically invalid cardiac shapes into close but correct shapes for introducing strong anatomical guarantees into the network. Khened et al. [15] proposed Densely Connected Fully Convolutional Network (DFCN), which is based on DenseNets [16]. Yang et al. [17] proposed a general and fully automatic solution to concurrently segment three important ventricular structures, starting from 3D Fully Convolutional Network (3D FCN). Simantiris and Tziritas [18] proposed a different Dilated CNN structure that incorporating domain-specific constraints. Isensee et al. [19] combined 2D U-Net and 3D U-Net, obtaining the best performance on the ACDC dataset. However, due to the combination of two different models, the numbers of model params is enormous. All these methods base on supervised learning proposed a series of efficient methods from different perspectives. When it comes to semisupervised cardiac MR image segmentation methods, there are still limitations for obtaining remarkable performance because cardiac MR image segmentation is a particular issue, including unique data distribution and difficult segmentation tasks.

### 2.2. Semisupervised Learning Methods

As for general semisupervised learning, many methods are proposed to reduce the burden of pixel-wise manual annotations for images, such as pseudo labeling [1], graph-based methods [20, 21], and entropy minimization [5]. Besides, mean-teacher [9] is another notable paradigm for semisupervised learning, which could be used in medical image segmentation. The mean-teacher model has two subnetworks: the teacher network and the student network, and learn cross-consistency from unlabeled data by exerting different perturbances on the two subnetworks. Yu et al. [22] proposed the uncertainty-aware mean teacher (UA-MT) framework, learning from the meaningful and reliable targets by exploiting the uncertainty information. Adversarial learning [23] methods are aimed at matching labeled and unlabeled images and improving testing time performance. Hung et al. [24] proposed a novel method in semisupervised semantic segmentation by introducing adversarial learning. Nie et al. [25] proposed attention-based semisupervised deep networks (ASDNet), where they integrated adversarial learning by a confidence network. Virtual Adversarial Training (VAT) [26] utilizes adversarial learning from a novel perspective and alters the model's predictions the most by approximating the perturbations. Laine and Aila [10] introduced consistency regularization into semisupervised learning, including *π*-model [10] and temporal ensembling method [10]. Bortsova et al. [27] proposed a novel semisupervised method that learns to predict segmentations consistent under a given class of transformations on both labeled and unlabeled images. The above methods enforce the consistency between predictions and provide critical data information to the supervised trained model. Besides, a series of strong data augmentation methods are proposed for overcoming the limitation of labeled training data, such as MixUp [28], CutMix [29], and Mosaic [30]. CowMix [31] starts from MixUp and enforces the consistency between the mixed outputs and the prediction over the mixed inputs. All the above data augmentation methods have made efforts to semisupervised learning by increasing training data diversity.

### 2.3. Lightweight Deep Networks

Current existing lightweight methods for networks can be divided into model compression and lightweight architecture design. We mainly review methods designing lightweight architectures, which are more related to our study. The increasing need to deploy deep models on computationally limited platforms and process large-scale data encourages lightweight architecture design. A series of lightweight convolutional modules have been proposed to balance the model performance and computational complexity. In particular, depth-wise convolution [32] and group convolution [33, 34] have gained much attention and have been building blocks for many lightweight architectures. MobileNet [35] used depth-wise separable convolution [32], a combination of depth-wise convolution and point-wise convolution, to build a lightweight model. ShuffleNet [36] is presented with point-wise group convolution and channel shuffle, which improves the information flow exchange between channel groups. Recently, Han et al. [11] proposed GhostNet with a novel Ghost module, which utilizes group convolution to further explore correlation and redundancy between feature maps. The GhostNet has shown higher recognition performance in natural images but has not been applied in medical image segmentation tasks.

## 3. Methods

### 3.1. Problem Formulation

We aim to develop a deep network model for semantic segmentation of cardiac MR images with only a few annotated subjects and a larger set of unlabeled subjects. We segment cardiac MR sequences in a slice-by-slice manner. Assume *𝒟*_*l*_ = {*X*^*l*^, *Y*^*l*^} denote the labeled data, in which *X*^*l*^ = {*x*_1_^*l*^, *x*_2_^*l*^, ⋯, *x*_*n*_^*l*^} contains *n* image slices, and *Y*^*l*^ = {*y*_1_^*l*^, *y*_2_^*l*^, ⋯, *y*_*n*_^*l*^} is ground truth. *𝒟*_*u*_ = {*x*_1_^*u*^, ⋯, *x*_*m*_^*u*^} denotes *m* unlabeled examples. Usually, the number of unlabeled slices is much larger than labeled ones (*m* ≫ *n*). Making better use of unlabeled data is a critical part of training a semisupervised segmentation network with better generalization ability on unseen data.

An overview of the proposed LCC-Net is demonstrated in Figure 1. We leverage the unlabeled data during supervised segmentation model learning and encourage segmentation consistency on all data under different perturbations with two unsupervised consistency losses. Our segmentation network is in encoder-decoder architecture. Specifically, the LCC-Net contains a shared encoder *E* and three independent decoders: the supervised decoder *D*_*S*_, the dropout decoder *D*_*D*_, and the noise decoder *D*_*N*_. The encoder *E* and the decoder *D*_*S*_ constitute the segmentation network *f*_*S*_ = *D*_*S*_∘*E*. While the supervised decoder  *D*_*S*_ is trained with the labeled data, the two auxiliary decoders are trained with both labeled data and unlabeled data.

We inject perturbations in both the feature space, i.e., the output of the feature encoder *E* and the input image space.

- For perturbations in the feature space, we use two perturbations: dropout perturbation *P*_*D*_ and noise perturbation *P*_*N*_. The dropout decoder *D*_*D*_ and noise decoder *D*_*N*_ are used to decode the two perturbed versions of features, respectively. We enforce the consistency of predictions between the supervised decoder  *D*_*S*_ and the auxiliary decoders *D*_*D*_ and *D*_*N*_ with unsupervised consistency losses. These two auxiliary decoders together with the encoder and feature perturbations constitute the two auxiliary networks *f*_*D*_ = *D*_*D*_∘*P*_*D*_∘*E* and *f*_*N*_ = *D*_*N*_∘*P*_*N*_∘*E*. In the experiments, we use Gaussian noises for the noise perturbation *P*_*N*_ and 10%-40% spatial random dropout for the dropout perturbation *P*_*D*_
- For perturbations in the image space, we use a stronger perturbation *P*_*C*_ to achieve better model robustness. Specifically, we exploit an adapted version of the Cutmix [29], as illustrated in Figure 2. Given two input images, we first split the images into four blocks of equal size. Then, we randomly exchange one or two blocks on the corresponding positions between the two images. When the two input images are labeled, the corresponding operations are also applied to their label images

We apply the cutting and mixing perturbation on both the labeled data and unlabeled data as a data augmentation to the original data. In addition to the (augmented) unlabeled data, we also feed the perturbed labeled data to the auxiliary networks and enforce cross-model consistency.

### 3.2. Supervised Training on Few Labeled Data

The segmentation network *f*_*S*_ = *D*_*S*_∘*E* is trained with the (augmented) labeled data using a cross-entropy- (CE-) based supervised loss. We also denote the augmented labeled data as *𝒟*_*l*_ ∪ *𝒟*_*l*_′, where *𝒟*_*l*_′ is generated by perturbing the images in *𝒟*_*l*_ using cutting and mixing *P*_*C*_.

(1) $$\begin{array}{c} L_{S}=\frac{1}{\left|D_{l}\cup D_{l}^{\prime }\right|}\underset{\left(x_{i},y_{i}\right)\in D_{l}\cup D_{l}^{\prime }}{\sum }l_{\text{CE}}\left(x_{i},y_{i}\right), \end{array}$$

where *l*_CE_ denotes the cross-entropy loss. The input image *x*_*i*_^*l*^ can be the original image and its perturbed version.

### 3.3. Unsupervised Cross-Consistency Training

As mentioned above, we enforce cross-model consistency between the predictions of the supervised decoder  *D*_*S*_ and the auxiliary decoders *D*_*D*_ and *D*_*N*_ with an unsupervised consistency loss. We denote the augmented unlabeled data as *𝒟*_*u*_ ∪ *𝒟*_*u*_′, where *𝒟*_*u*_′ is generated by perturbing the images in *𝒟*_*u*_ using cutting and mixing *P*_*C*_. The two auxiliary networks *f*_*D*_ and *f*_*N*_ take both the (augmented) unlabeled data *𝒟*_*u*_ ∪ *𝒟*_*u*_′ and the perturbed labeled data *𝒟*_*l*_′. The two auxiliary networks are trained with the following loss.

(2) $$\begin{array}{c} L_{U}=\frac{1}{\left|D_{u}\cup D_{u}^{\prime }\cup D_{l}^{\prime }\right|}\underset{\left(x_{i},y_{i}\right)\in D_{u}\cup D_{u}^{\prime }\cup D_{l}^{\prime }}{\sum }\left[d\left(f_{S}\left(x_{i}\right),f_{D}\left(x_{i}\right)\right)+d\left(f_{S}\left(x_{i}\right),f_{N}\left(x_{i}\right)\right)\right], \end{array}$$

where the distance measure **d** is used to measure the consistency of the predictions by different models. In the experiments, we use mean squared error (MSE) as the distance measure.

### 3.4. The Overall Loss

By integrating the supervised loss and unsupervised loss, the loss of our LCC-Net reads

(3) $$\begin{array}{c} L=L_{S}+\lambda L_{U}, \end{array}$$

in which *λ* is the trade-off parameter. In the experiments, we choose an exp-schedule function as follows:

(4) $$\begin{array}{c} \lambda \left(\text{epoch}\right)=\min\left(\lambda_{\max},\lambda_{\max}\times e^{2\cdot \left(\text{epoch}/\text{stop}-1\right)}\right), \end{array}$$

in which epoch as current training epoch, stop is the max number of epochs to stop increasing *λ*, and *λ*_max_ is an upbound of *λ*.

### 3.5. The Backbone of the LCC-Net

To avoid overfitting on the small labeled data, we introduce a lightweight segmentation U-Net (L-Unet) as our backbone network, which is demonstrated in Figure 3. The network is an encoder-decoder with skip-connections between the corresponding layers of the encoder and decoder. To lighten the U-Net, we upgrade the U-Net with lightweight convolutional modules. More precisely, we replace the standard convolutions in U-Net with the Ghost module [11], which involves much fewer parameters and computation costs. The Ghost module is shown in Figure 4. For a feature map *F* ∈ ℝ^*a*×*h*×*w*^, in which *a* is the channel number, and *h* × *w* is the spatial size, we first compress *F* into *F*′ ∈ ℝ^(*b*/*s*)×*h*×*w*^ by using a standard 3 × 3 convolution, where *b* is the channel number of the final output, and *s* is the ratio. Then, we apply *s*(=4) linear transformations, including one identity transform, on each channel of *F*′ separately to generate *s* groups of new features, each of which contains *b*/*s* feature maps. The linear transformations are achieved with 3 × 3 convolutions. At last, we concatenate all the generate feature maps and obtain the final output $\hat{F}\in {\mathbb{R}}^{b\times h\times w}$. Note that the computation costs of the linear transformations are much lower than standard convolutions. The model size of the L-Unet is only 8.7 M, which is four times less than that of the U-Net (35.5 M).

## 4. Experiments and Results

In this section, we conduct a series of experiments to evaluate the proposed LCC-Net's performance for semisupervised cardiac segmentation.

### 4.1. Dataset and Evaluation Measure

*ACDC Dataset*. We first utilize ACDC (Automated Cardiac Diagnosis Challenge) [12] dataset in our experiments, which belongs to a cardiac MR images segmentation challenge in MICCAI 2017. The ACDC dataset includes the short-axis cine-MRI of 150 subjects acquired from the University Hospital of Dijon using two MR scanners of different magnetic strengths. Left ventricle (LV), right ventricle (RV), and myocardium (MYO) were manually annotated by clinical experts on end-diastolic (ED) and end-systolic (ES) phase instants. The organizer of the ACDC splits the whole dataset into two subsets: (1) 100 subjects with available ground truth and (2) 50 subjects without ground truth for online testing.

We use the 100 labeled subjects (including 1902 image slices) for model evaluation. We randomly selected 20 subjects (containing 380 slices) as the testing set. The remaining 80 subjects are used as the union of the labeled data and unlabeled data. Specifically, we randomly select *K* subjects (2, 4, 6, and 10) for model training and the remaining 80- *K* subjects as the unlabeled data.

*Evaluation Criteria*. Our experiments utilize the Dice Coefficient (DICE) and Hausdorff distance (HD) as the evaluation criteria. Given the ground truth *X* and the prediction *Y*, DICE, which evaluates the region overlap of different segmentations, is defined as

(5) $$\begin{array}{c} \text{DICE}=\frac{2∙\left|X\cap Y\right|}{\left|X\cup Y\right|}. \end{array}$$

The HD is defined as

(6) $$\begin{array}{c} \text{HD}\left(X,Y\right)=\max\left\{\underset{a\in X}{\max}E\left(a,Y\right),\underset{b\in Y}{\max}E\left(b,X\right)\right\}, \end{array}$$

where *E*(*a*, *X*) is the Euclid distance between *a* and *X*.

### 4.2. Implementation Details

We implemented our experiments on the framework of PyTorch [37] on one GTX 1080 GPU with 8 G memory. We used the adaptive moment estimation (Adam) optimizer with the learning rate of 5 × 10^−4^ initially, decreasing by 0.5 in epochs 200, 1000, 1500, 1800, and 2100. Moreover, the batch size was set as 4 because of the limitation of the GPU. The maximum epochs of iterations were set as 3000, and *λ*_max_ was set as 0.4. Data augmentation, including affine transform, random rotation, and random intensity shift, was used. All the images were resized to 160 × 160, and the intensity range of each image was rescaled to [0, 1].

### 4.3. Segmentation Performance

#### 4.3.1. Comparative Results of the LCC-Net

We first conduct a comparative study to identify the effectiveness of the critical components in the proposed model, including the backbone network L-Unet, the dropout decoder *D*_*D*_, the noise decoder *D*_*N*_, and the input space perturbation *P*_*C*_. Specifically, we randomly select *K* = 2 subjects (40 slices) as the labeled data and the remaining 78 subjects as the unlabeled data, which are used for model training.

Table 1 summarizes the results of the comparative studies. The results of 7 network and data settings are reported: (1) the upbound, i.e., the U-Net trained with all the 80 labeled data; (2) the U-Net as the baseline, which is trained from scratch using the labeled data with standard data augmentations; (3) the L-Unet, which is also trained from scratch using the labeled data with standard data augmentations; (4) the LCC-Net w/o *P*_*C*_, which is trained on both the labeled and unlabeled data without the input space perturbation *P*_*C*_; (5) the LCC-Net w/o *P*_*N*_, which is trained on both the labeled and unlabeled data without the noise decoder *D*_*N*_; (6) the LCC-Net w/o *P*_*D*_, which the LCC-Net without the dropout decoder *D*_*D*_; (7) the full LCC-Net.

As shown in Table 1, when training with only two labeled subjects, the U-Net has a mean performance drop of 32.7% in DICE and 9.2 mm in Hausdorff than the U-Net trained with 80 subjects. Rather than using more labeled data, we exploit the unlabeled data, which is much easier to collect. As illustrated in Table 1, by exploiting unlabeled data, the LCC-Net outperforms the U-Net (baseline) by a large margin, i.e., 14.4% in the mean DICE and 4.3 mm in the mean Hausdorff over the three regions. LCC-Net without using the noise perturbation *P*_*N*_ and noise decoder *D*_*N*_ obtains a performance gain of 12.2% in DICE and 5.9 mm in Hausdorff over the L-Unet; LCC-Net without using the dropout perturbation *P*_*D*_ and dropout decoder *D*_*D*_ obtains a performance gain of 13.4% in DICE and 6.1 mm in Hausdorff over the L-Unet. Compared to the full LCC-Net, the LCC-Net without using the input space perturbation *P*_*C*_ shows a mean performance drop of 4.4% in DICE and 3.2 mm in Hausdorff, which indicates the effectiveness of the input space perturbation *P*_*C*_. However, with only two labeled subjects for model training, the semisupervised model's performance is still significantly lower than the fully supervised U-Net.  Figure 5 provides a visual comparison of the LCC-Net without *P*_*N*_, LCC-Net without *P*_*D*_, and our LCC-Net. Visually, the LCC-Net shows significantly better results than the other two methods.

#### 4.3.2. The Impact of the Number of the Labeled Subjects

Since our method is a semisupervised method, it is crucial to identify the impact of the size of the labeled training dataset. To this end, we trained our model with different choices of *K*, i.e., 2, 4, 6, and 10 subjects.  Table 2 summarizes the experimental results. The results with U-Net under different settings, including the fully supervised setting (80 labeled subjects), are also reported. As can be expected, with increasingly more labeled data for model training, the performance becomes much higher. With the different choices of *K*, our semisupervised model consistently outperforms the U-Net. Remarkably, using only four labeled subjects, our model outperforms the U-Net trained on ten labeled subjects. Using ten labeled subjects for training, the LCC-Net achieves a mean performance of 82.4%, which is 6.1% higher in mean DICE than the U-Net.  Figure 6 demonstrates a further comparison of the proposed model and the U-Net, which shows the effectiveness of our model.

#### 4.3.3. The Impact of the Selection of the Labeled Subjects

To identify the robustness of the proposed model over the different selections of the label data. To this end, we randomly selected five samples and calculated the mean performance and the standard variance. Here, each sample contains two subjects as the labeled data. The results are reported in Table 3. Although each sample size is very small (2 subjects), our model shows relatively stable performance.

### 4.4. Model Complexity

Model complexity is typically measured by the number of trainable network parameters (i.e., model size) and the floating-point operations (FLOPs). The model complexity of our model is summarized in Table 4. Our model obtained significantly reduced model size and FLOPs at both the training stage and testing stage by replacing standard convolutions with the lightweight module. Therefore, our model requires less computation cost for each training step and inference step, resulting in higher computational efficiency. The inference time at the testing stage is a critical measure in practical usage. As shown in Table 4, with reduced FLOPs, the proposed LCC-Net involves a shorter inference time than the LCC-Net using standard convolutions.

## 5. Conclusion

In this paper, we presented a lightweight cross-consistent network for semisupervised cardiac MR image segmentation. We leveraged the unlabeled data during supervised segmentation model learning and encourage segmentation consistency on all data under different perturbations with two unsupervised consistency losses. To achieve a lightweight model, we replaced the standard convolutions with a lightweight module. Extensive comparison experiments with a public dataset demonstrated that our architecture achieved promising performance with only two labeled subjects.

Despite the improved results, there are still more applicable perturbations in semisupervised segmentation. Thus, exploring more efficient perturbations is a significant work in the future.

## Figures and Tables

**Figure 1:** Overview of our LCC-Net for semisupervised segmentation. The network contains one supervised decoder and two unsupervised decoders. While the supervised decoder is trained with the labeled data, the two auxiliary decoders are trained with both labeled data and unlabeled data using unsupervised consistency losses. We inject dropout perturbation and noise perturbation in the feature space and inject cutting and mixing perturbation in the input image space.

**Figure 2:** Illustration of the input space perturbation *P*_*C*_ used in our study. (a) The cardiac MR images. From left to right: original image A, original image B, the perturbed image *A*′, and the perturbed image *B*′. (b) Their corresponding label images. We evenly split an image into four blocks and then randomly exchange one or two blocks on the corresponding positions. The same operations are applied on their ground truth label images, as in (b). Best view in color.

**Figure 3:** The backbone network of our proposed model, L-Unet. Instead of standard 2D convolutions, the L-Unet uses the Ghost module [11] as the basic building block.

**Figure 4:** The architecture of Ghost module [11], which uses a series of cheap transformation operations to generate ghost feature maps, which results in significantly reduced computational complexity.

**Figure 5:** Visualization of the performance of the ablated versions of our LCC-Net.

**Figure 6:** The impact of the number of the labeled subjects.

**Table 1:** Comparative study of the proposed LCC-Net on the ACDC dataset. We randomly selected 2 subjects as the labeled data and the remaining 78 subjects as the unlabeled data. The models are tested on 20 unseen subjects. *P*_*C*_ denotes the perturbations in the feature space, *P*_*N*_ denotes the noise perturbation in the feature space, and *P*_*D*_ denotes the dropout perturbation in the feature space.

Method	Labeled data	DICE (%)				Hausdorff (mm)			
		LV	RV	MYO	Mean	LV	RV	MYO	Mean
U-Net (upbound)	80 subjects	93.2	85.8	88.9	89.3	2.2	4.8	2.8	3.3
U-Net (baseline)	2 subjects	76.1	24.7	69.1	56.6	9.2	17.0	11.4	12.5
L-Unet		69.9	36.7	60.2	55.6	10.7	19.2	12.7	14.2
LCC-Net w/o *P*_*C*_		78.2	52.0	69.6	66.6	7.8	16.6	9.8	11.4
LCC-Net w/o *P*_*N*_		78.0	54.8	70.7	67.8	5.8	11.3	7.8	8.3
LCC-Net w/o *P*_*D*_		80.6	53.6	73.0	69.0	5.6	11.9	6.9	8.1
LCC-Net		82.0	58.1	73.0	71.0	4.3	13.9	6.3	8.2

**Table 2:** The impact of the number of the labeled subjects. The results are tested on the ACDC dataset.

Labeled data	Method	LV (%)	RV (%)	MYO (%)	Mean (%)
2 subjects	U-Net (baseline)	76.1	24.7	69.1	56.6
	LCC-Net	82.0	58.1	73.0	71.0
4 subjects	U-Net (baseline)	79.6	51.7	71.1	67.5
	LCC-Net	85.0	69.3	76.9	77.1
6 subjects	U-Net (baseline)	83.4	62.3	74.0	73.2
	LCC-Net	85.0	74.5	79.3	79.6
10 subjects	U-Net (baseline)	82.1	70.1	76.6	76.3
	LCC-Net	87.4	77.0	82.8	82.4
Fully supervised (80 subjects)	U-Net (baseline)	93.2	85.8	88.9	89.3

**Table 3:** The impact of the selection of the labeled subjects. The results are tested on ACDC dataset. Five samples are randomly selected, where each sample contains two labeled subjects as the labeled data for model training.

	DICE (%)							Hausdorff (mm)						
	(1)	(2)	(3)	(4)	(5)	Mean	Std	(1)	(2)	(3)	(4)	(5)	Mean	Std
LV	82.0	83.6	78.8	80.8	82.1	81.5	1.6	4.3	4.5	6.8	5.6	5.3	5.3	0.9
RV	58.1	64.0	51.0	52.9	54.6	56.1	4.6	13.9	9.1	12.4	11.9	10.1	11.5	1.7
MYO	73.0	74.1	73.6	73.9	75.5	74.0	0.8	6.3	5.8	6. 7	6.4	5.6	6.2	0.4
Mean	71.0	73.9	67.8	69.2	70.7	70.5	2.0	8.2	6.5	8.6	8.0	7.0	7.7	0. 8

**Table 4:** A comparison of the model complexity of the LCC-Net with different building blocks. The total inference time denotes the inference time on the whole testing set (402 images of 160 × 160).

LCC-Net with	Model size		FLOPs		Total
	Training	Testing	Training	Testing	Inference time
Standard convolution	81.5 M	35.5 M	329.8 G	102.8 G	20.8 s
Ghost module (*s* = 4)	25.2 M	8.7 M	91.0 G	26.2 G	17.3 s

## Data Availability

The data used in our experiments are available at https://www.creatis.insa-lyon.fr/Challenge/acdc/.
